# A Study of Racket Weight Adaptation in Advanced and Beginner Badminton Players

**DOI:** 10.1155/2024/8908294

**Published:** 2024-01-25

**Authors:** Zhengye Pan, Lushuai Liu, Xingman Li, Yunchao Ma

**Affiliations:** College of Physical Education and Sports, Beijing Normal University, Beijing, China

## Abstract

The jump smash is the most aggressive manoeuvre in badminton. Racket parameters may be the key factor affecting the performance of jump smash. Previous studies have focused only on the biomechanical characteristics of athletes or on racket parameters in isolation, with less observation of the overall performance of the human-racket system. This study aims to explore the effects of different racket weights on neuromuscular control strategies in advanced and beginner players. Nonnegative matrix factorisation (NMF) was used to extract the muscle synergies of players when jumping smash using different rackets (3U, 5U), and K-means clustering was used to obtain the fundamental synergies. Uncontrolled manifold (UCM) analyses were used to establish links between synergy and motor performance, and surface electromyography (sEMG) was mapped to each spinal cord segment. The study found significant differences (*P*  < 0.05) in the postural muscles of skilled players and significant differences (*P*  < 0.001) in the upper-limb muscles of beginners when the racket weight was increased. Advanced players adapt to the increase in racket weight primarily by adjusting the timing of the activation of the third synergy. Combined synergy in advanced players is mainly focused on the backswing, while that in beginners is mainly focused on the frontswing. This suggests that advanced players may be more adept at utilising the postural muscles and their coordination with the upper-limb muscles to adapt to different rackets. In addition, the motor experience can help athletes adapt more quickly to heavier rackets, and this adaptation occurs primarily by adjusting the temporal phase and covariation characteristics of the synergies rather than by increasing the number of synergies.

## 1. Introduction

In badminton, the forehand jump smash is usually the most aggressive stroke. By synergistically activating the postural muscles with the upper-limb muscles, the jump smash allows for a faster smash, a higher contact point, and a steeper shot, making it more difficult for the opponent to return as it gives them less time to retrieve the shuttlecock [1]. In addition to the requirement for good neuromuscular control strategies during the jump smash, the racket is also a key factor influencing the performance of the human-racket system, which indirectly affects the score [2]. Most of the studies on the jump smash have focused exclusively on the kinematic, kinetic, or muscle activation characteristics of the body, with a relatively large number of studies on elite athletes in particular [3, 4], and all of the studies on the racket have tended to focus on the racket in isolation and have not taken into account the athlete's use of the racket [5]. In other words, fewer studies have focused on the effects of different rackets on motor performance, especially on neuromuscular activation strategies.

Some studies have found that long-term training can optimise the neuromuscular control strategies required to accomplish high-quality performance [6]. Motor experience can motivate the central nervous system (CNS) to choose more stable, low-cost control strategies for high-quality manoeuvres in the face of substantial redundancy in the musculoskeletal system. Matsunaga and Kaneoka [7]. compared the differences in muscle synergies between elite and no-elite athletes during jump smash and found that the number of synergies in elite athletes was one more than in no-elite athletes. Muscle synergy refers to the phenomenon that the CNS controls movement through fewer core variables rather than individual muscles [8, 9]. This suggests that long-term training promotes the creation of a new synergy that is more specific to the manoeuvre. However, the study did not further analyse the covariation properties of the synergies to establish a link between muscle synergies and performance, which left the study isolated at the muscle level.

The aim of this study was to investigate the effects of different racket weights on neuromuscular activation strategies in advanced and beginner players and to attempt to further establish a link between performance and muscle synergy. sEMG and kinematic data were collected from skilled and beginner players when jumping smash with different rackets (3U, 5U). Muscle synergy was extracted using NMF, and the combined synergy was further separated from the fundamental synergy using the K-means algorithm to avoid its interference with the fundamental synergy. UCM analysis was used to establish the link between each synergy and shoulder internal rotation and to explore the covariation properties of synergies in different kinds of subjects in maintaining shoulder stability (low-variability). In addition, sEMG was mapped to spinal cord segments to assess their motor output and to analyse the extent to which upper-limb muscles and postural muscles were utilised by subjects of different levels when using different rackets.

## 2. Materials and Methods

### 2.1. Participants

The sample size was determined using *G* ^*∗*^ power (v3.1.9.2, Heinrich-Heine University, Düsseldorf, Germany) based on the previous study [10] (*α* = 0.05, power = 80%). Based on the subject selection criteria of previous study [7], nine male advanced badminton players with more than 7 years of training were recruited as the high-level group, and nine male beginner players with less than 1 year of training were recruited as the low-level group. The comparison of the characteristics of the two groups of subjects is shown in Table 1. To assess the adaptability of different levels of subjects to different rackets, these subjects were asked to have 4U as their usual racket. A professional badminton coach was responsible for the selection of the subjects. All subjects were required to be free of neuromuscular and musculoskeletal injuries as well as head or spinal cord injuries within 6 months, with the right hand as the dominant hand.

### 2.2. Data Collection

All data were collected on a full-size standard badminton court to avoid the effects of the laboratory environment on the subjects. Kinematic data were acquired using a Vicon 3D motion capture system (200 Hz, V5, Oxford, UK; 8 cameras, 14 mm reflective markers). The Marker protocol was set with reference to the previous study [11], in which the markers for the upper limbs were set as shown in Table 2. In order to minimise input resistance and external interference, some preparations were made before acquiring the sEMG, including shaving and cleaning the skin surface. The sEMG signals of 13 muscles of the trunk and right upper limb were acquired using a Delsys wireless sEMG tester (2,000 Hz, Trigno, Boston, USA) [1, 12]: Brachioradialis (BR), Extensor digitorum (ED), Flexor carpi ulnaris (FC), Biceps brachii (BI), Triceps brachii (TR), Anterior Deltoid Front (ADF), Posterior Deltoid Rear (PDR), Latissimus dorsi (LA), Trapezius (TR), Pectoralis Major (PM), Rectus abdominis (RA), External oblique (EO), and Erector spinae (ES).

New Yonex Aerosense 30 shuttlecocks (Yonex, Tokyo, Japan) with a circle of reflective tape (diameter 16 mm) attached to the tip of the shuttlecock were used for the data collection. Shuttlecocks that were misshaped or broken were discarded. All subjects used the same standard 3U and 5U badminton racket. All participants were given approximately 15 min to warm up and 15 min to familiarise themselves with the environment. During data collection, a badminton trainer threw shuttlecocks from a fixed position. To avoid the effect of different angles on the muscle synergy of the subjects, the optimal jumping smash angle was self-selected by the subjects during the warm-up [13]. Each subject was required to complete five jump smashes successfully, with a 2-min rest period between each trial.

### 2.3. Data Analysis

Computing generalised kinematic characteristics with Visual3D (C-Motion Inc., Germantown, USA) and obtaining three key frames: preparation (most flexed knee angle before the push-off), racket lowest point (RLP) defined as the lowest vertical height of the racket tip marker between preparation and shuttle–racket contact, and shuttle–racket contact (frame where the anterior–posterior velocity of the shuttlecock changes from negative to positive) [2]. Based on these three frames, the jump smash is divided into two phases: the backswing phase from the preparation to the RLP, and the frontswing phase from the RLP to the shuttle–racket contact. The backswing phase and the frontswing phase were normalised to 100%, respectively.

The filter cut-off frequency for the kinematic data was calculated according to the residual algorithm proposed by Giakas and Baltzopoulos [14]. The raw sEMG signals were high-pass filtered (50 Hz, 4th-order IIR), full-wave rectified, and low-pass filtered (20 Hz, 4th-order IIR) and a linear envelope constructed based on Python (v3.9.13, Delaware, US), followed by amplitude normalisation based on maximum activation [15].

#### 2.3.1. Spinal Motor Output Assessment

To describe the spinal motor output pattern, 13 sEMG signals collected were mapped to the rostrocaudal location of the pool of alpha-motor neurones (MNs) in the cervical vertebras (*C*_2–8_), thoracic vertebras (T_1_, T_12_) and a lumbar vertebra (L_1_). The cervical segment mainly innervates the muscles of the upper limbs, the thoracic and lumbar segments mainly innervate the postural muscles. The contribution of each muscle to the integrated activity of the spinal cord segments was calculated using the neuromuscular map proposed by Kendall et al. [16]. The motor output of each spinal cord segment *S*_*j*_ was estimated using the following equation, assuming a common spinal topography among subjects:

(1) $$\begin{array}{c} S_{j}=\frac{\sum_{i=1}^{m_{j}}\left(\frac{k_{ji}}{n_{i}}\times {\text{EMG}}_{i}\right)}{\sum_{i=1}^{m_{j}}\left(\frac{k_{ji}}{n_{i}}\right)}, \end{array}$$

where *m*_*j*_ is the muscle innervated by each spinal cord segment, *n*_*i*_ is the number of spinal cord segments innervating *i*th muscle, and *k*_*ij*_ is the weight of each muscle relative to the innervated spinal cord segment [17].

#### 2.3.2. Muscle Synergy Extraction and Geometrisation of Motor Primitives

Muscle synergies were extracted using a classical Gaussian NMF algorithm based on R (v4.2.2, Vienna, Austria). A matrix *V* was constructed with muscle activity patterns (*m* = 13) and normalised time points (*n* = 200) as rows and columns, respectively, and *V* was reconstructed into V_*r*_ by NMF as follows:

(2) $$\begin{array}{c} V\approx V_{r}=MP, \end{array}$$

where *r* is the number of synergies extracted. *M* is the motor module (*m* × *r*) and *P* is the motor primitive (*r* × *n*). The motor module describes the relative weights of each muscle in the *r* synergies, and the motor primitive describes the time-varying characteristics of the *r* synergies controlled by the CNS. The EM algorithm was used to iteratively update to obtain the optimal number of synergies:

(3) $$\begin{array}{c} \left\{\begin{array}{c} P_{i+1}=P_{i}\frac{M_{i}^{T}V}{M_{i}^{T}VM_{i}P_{i}}\\ M_{i+1}=M_{i}\frac{V{\left(P_{i+1}\right)}^{T}}{M_{i}P_{i+1}{\left(P_{i+1}\right)}^{T}} \end{array}\right.. \end{array}$$

Reconstruction quality was assessed by calculating the coefficient of determination (*R*^2^) between *V* and V_*r*_. Convergence was reached when the change in *R*^2^ was less than 0.01% in the last 20 iterations [15]. Clustering was performed based on the number of synergies per subject using the K-means algorithm with mean-squared error (MSE) as the loss function, and the optimal number of synergies, *r*, was obtained when the MSE was less than 10^−4^ [18]. The synergy that emerges from dimensionality reduction, which is composed of multiple fundamental synergies together, is defined as a combined synergy.

The centre of activity (CoA) was used to calculate the temporal phase of activation for motor primitives [19] as follows:

(4) $$\begin{array}{c} \left\{\begin{array}{c} A=\sum_{t=1}^{p}\left(\text{cos }\theta_{t}\times P_{t}\right)\\ B=\sum_{t=1}^{p}\left(\text{sin }\theta_{t}\times P_{t}\right)\\ \text{CoA}=\text{arctan }\left(B/A\right) \end{array}\right., \end{array}$$

where *p* is the time point of the normalised motor task. The full-width at half-maximum (FWHM) was used to describe the activation intensity of motor primitives [20].

#### 2.3.3. Uncontrolled Manifold Analysis

The UCM analysis [21] assumes that the CNS manipulates a set of elemental or controlled variables and tries to limit their variance to a subspace corresponding to a desired value of a performance variable. According to the previous studies, shoulder internal rotation is the most critical kinematic variable in jump smash. Therefore, shoulder internal rotation in this study was used as a performance variable in UCM analysis. We further followed a control hypothesis of Krishnan et al. [22]: CNS can maintain low variability in the kinematics variables by promoting the covariation of muscle synergies. Therefore, the *r* muscle synergies extracted above were used as elemental variables, and the shoulder internal rotation was used as the performance variable. Linear relationships between the controlled and performance variables were established using multiple regression coefficients [22]:

(5) $$\begin{array}{c} \sum_{i=1}^{r}n_{i}{\Delta \text{Syn}}_{i}=\Delta \theta_{\text{shoulder}}, \end{array}$$

where *n* is the regression coefficient, *r* is the number of synergies, and ΔSyn_*i*_ is the fluctuation of each synergy around the mean value across all subjects. The UCM can be approximated as the zero-space N(J) of the Jacobi matrix J of the regression coefficients, and the UCM is calculated from the zero-space basis *ε*_*i*_^*T*^ of J as follows:

(6) $$\begin{array}{c} \left\{\begin{array}{c} f_{\text{UCM}}=\sum_{i=1}^{r-d}{\left(\varepsilon_{i}^{T}\cdot \Delta \text{Syn}\right)}^{T}\cdot \varepsilon_{i}^{T}\\ f_{\text{ORT}}=\Delta \text{Syn}-{\left(f_{\text{UCM}}\right)}^{T} \end{array}\right., \end{array}$$

where *d* is the number of performance variables. To calculate the UCM and ORT variance across subjects:

(7) $$\begin{array}{c} \left\{\begin{array}{c} V_{\text{UCM}}=\frac{1}{\left(r-d\right)N}\sum_{i=1}^{N}f_{\text{UCM}}^{2}\\ V_{\text{ORT}}=\frac{1}{N}\sum_{i=1}^{N}f_{\text{ORT}}^{2}\\ V_{\text{TOT}}=\frac{1}{\left(r+d\right)N}\sum_{i=1}^{N}{\left(\Delta \text{Syn}\right)}^{2} \end{array}\right., \end{array}$$

where *N* is the number of subjects. The synergy index *ΔV* is used to quantify the strength of the covariation in the synergies to stabilise the *θ*_shoulder_, and the Fisher *z*-transform is used to correct *ΔV* for a normal distribution [23]:

(8) $$\begin{array}{c} \left\{\begin{array}{c} \Delta V=\frac{V_{\text{UCM}}-V_{\text{ORT}}}{V_{\text{TOT}}}\\ \Delta V_{z}=\frac{1}{2}\text{log}\left[\frac{\left(r+d\right)+\Delta V}{\frac{r+d}{r-d}-\Delta V}\right] \end{array}\right.. \end{array}$$

The larger the value of *ΔV_z_*, the greater the ability of the synergies to collaborate to stabilise the variability of the *θ*_shoulder_.

### 2.4. Statistical Analysis

The Shapiro–Wilk (SW) test was used to test for normal distribution, and the Mauchly sphericity test was used to test whether the sphericity hypothesis is met, and two-way repeated measures ANOVA was used to compare the spinal motor output *S*_j_, CoA, and synergy index with a Bonferroni post hoc test. One-dimensional statistical parametric mapping (SPM1d) based on a two-way repeated measures ANOVA was used to compare the differences of motor primitives between advanced and beginner players. All significance levels were set at 0.05, and statistical analysis is based on Python (https://spm1d.org/).

## 3. Results

### 3.1. Spinal Motor Output

Figure 1 shows the characteristics of the spatial and temporal distribution of spinal motor output in different subjects using 3U and 5U for jump smash. Significant differences (*P*  < 0.05) were found in the segments (T_1_, T_12_, and L_1_) that innervate the postural muscles, including the erector spinae, rectus abdominis, and external abdominal obliques, in skilled subjects when using different rackets. In contrast, there was a significant difference in the C_2_–C_5_ segments of the beginner players when using different rackets, which predominantly innervate the shoulder and elbow muscles such as the brachioradialis, biceps, triceps, deltoid, and trapezius muscles (*P*  < 0.001).

### 3.2. Muscle Synergy Characteristics

The NMF reduction parameters for different levels of subjects are shown in Table 3. The quality of reconstruction for muscle synergy was significantly higher in advanced players than in the beginner players (*P*  < 0.05). In addition, the percentage of combined synergy was lower in advanced players than in the beginner players.

The muscle synergy characteristics of the subjects at different levels are shown in Figure 2. Both advanced and beginner players have four muscle synergies when using different rackets. The first synergy is mainly located in the initial backswing phase and is dominated by the muscles around the elbow and wrist, which are mainly responsible for completing the preparatory action of the shot. The second synergy is mainly distributed in the mid-end backswing, which involves the activation of the postural muscles (especially the rectus abdominis) in addition to the upper-limb muscles, further increasing the potential energy reserve. The third synergy is distributed in the initial-mid frontswing phase and involves a substantial activation of the elbow extensors to increase the angular velocity of the end of the limb during the jump smash. The fourth synergy is distributed in the end frontswing and involves extensive activation of the postural muscles to improve postural stability before landing.

In addition, there was a significant difference in the third synergy between 3U and 5U for advanced players (*P*  < 0.001; 120%–160%). Compared with beginners, advanced subjects with the 3U exhibited slower second synergy activation (*P*  < 0.001; 100%–117%). Similarly, both the second synergy (*P*  < 0.001; 95%–130%) and third synergy (*P*  < 0.001; 145%–170%) in beginners were significantly different from skilled subjects when using the 5U.

### 3.3. Geometrisation Characteristics of Motor Primitives

The geometrisation characteristics of the motor primitives of the subjects at different levels are shown in Figure 3. The main distribution of combined synergies in advanced subjects was concentrated in the backswing phase, whereas the distribution of combined synergies in beginners was concentrated in the frontswing phase (*P*  < 0.05). The degree of concentration of each synergy when using 3U was significantly higher in the advanced players than in the beginners (*P*  < 0.05). The activation phases of synergy 2–4 were all earlier in beginners compared to the skilled players (*P*  < 0.05), but there was no significant difference in the strength of activation of synergy between the two groups of subjects.

### 3.4. UCM Analysis

Figure 4 shows the characteristics of the synergy index for subjects at different levels. When using the 3U racket, the synergy index was significantly greater in advanced subjects than in beginners during the backswing phase (*P* < 0.001) and significantly less during the frontswing phase (*P* < 0.001). In addition, both advanced and beginner players exhibited anticipatory synergy adjustments (ASAs) in the synergy index before the contact point, but there was no significant difference in the rate of adjustment between the two types of subjects.

## 4. Discussion

This study used a combination of machine learning and NMF to explore the adaptation of different rackets during jump smash in subjects of different levels, and further used UCM analysis to establish a link between muscle synergy and motor performance. The present study found that when racket weight was changed, skilled players tended to avoid the effects of racket weight changes on motor performance by changing the control strategy of the postural muscles rather than the upper-limb muscles, which is contrary to the beginner players. In fact, in many sports, athletes with extensive motor experience are usually more adept at responding to changes in motor conditions by adjusting the activation of their core muscles to ensure high-quality performance [24]. For example, experienced footballers performing side-step cutting at different angles can enhance the aggressiveness of the manoeuvre by flexibly adjusting the coordinated activation of the postural and lower-limb muscles [25]. This finding suggests that more attention should be paid to the exercise of the postural muscles in the daily training of badminton. In addition, advanced subjects showed stronger activation of the postural muscles in both the backswing and frontswing compared to beginner players, which is consistent with the findings of Pardiwala et al. [26]. The postural muscles are not activated for the same purpose in the two phases: in the backswing phase they are mainly used to enhance the aggressiveness of the jump smash, whereas in the frontswing phase they are mainly used to enhance postural stability before landing. This potentially supports the findings of previous studies that motor experience can motivate the CNS to select more adaptive control strategies to optimise motor performance [25].

In this study, it was found that the muscle activation patterns of both advanced and beginner players during jump smash using different rackets could be indicated by four synergies. This is contrary to the previous findings [7] that skilled subjects can differentiate specific muscle synergy in response to jumping smash. Indeed, there has been controversy regarding the effect of motor experience on muscle synergy in the jumping smash, and a study by Barnamehei et al. [10] found no significant difference in muscle synergy between advanced and beginner players during the jumping smash. Although, the number of synergies was the same for both advanced and beginner players in this study, advanced subjects were able to adapt to the increase in racket weight by adjusting the timing of activation of the third synergy, whereas beginners did not have this ability. This suggests that the optimising effect of motor experience is specifically demonstrated by the possibility of facilitating the adjustment of the temporal phases of synergy activation, which ensures high-quality motor performance. In addition, the percentage of combined synergy was lower in skilled subjects compared to beginners and was concentrated in the backswing phase. Although, the present study did not investigate combined synergy in-depth, previous studies have found that this combined synergy, formed by combining multiple fundamental synergy, is similar to the impaired synergy, often leads to an increase in muscle activity and energy expenditure, which may be the main reason for sports injuries, and is often used as an evaluation index for assessing the risk of sports injuries [8, 27, 28]. This suggests that an increase in racket weight may increase the risk of sports injuries and that injuries in advanced players are more likely to occur in the backswing phase.

In the investigation of synergy indices, this study found that both advanced and beginner players showed ASAs when jumping smash using the 3U, and that ASAs were earlier in advanced players than in beginners. Krishnan et al. [22] argued that ASAs reflect the fact that the degree of covariation between control variables can be prepared for subsequent rapid changes in the performance variables by attenuating them in advance. Recent research has suggested that ASAs represent the superposition of two processes: the ASAs with minimal net mechanical effects and the generation of forces/moments that resist the expected perturbations [29, 30]. The results of this study suggest that an increase in racket weight can contribute to the emergence of ASAs and that motor experience can help players adapt more quickly to the effects of increased racket weight.

There are certain limitations to this study. Despite the preestimation of the sample size in this study, subjects may be affected by different teaching methods or sports training, which in turn affects muscle synergy in both groups of subjects, and therefore further expansion of the sample size is needed in subsequent studies. In addition, only male subjects were recruited in this study, and the effect of gender differences in the process of motor adaptation was not considered and will be explored in the subsequent studies.

## 5. Conclusions

Advanced players responded to changes in racket weight primarily by adjusting activation strategies in the postural muscles, whereas beginners responded by adjusting activation strategies in the upper-limb muscles. Motor experience does not affect the number of muscle synergies during the jump smash, but it can be used to increase adaptation by improving the temporal phase of activation of synergies and by adjusting the covariation characteristics of synergies. Additionally, advanced players may suffer injuries during the backswing phase when using a heavier racket, whereas beginners may suffer injuries during the frontswing phase.

## Figures and Tables

**Figure 1:** Characteristics of spatial and temporal distribution of spinal motor output during jump smash in different subjects. The horizontal axis is backswing and frontswing phase normalised to 100%, and the vertical axis is alpha-motor neurone activity in 12 spinal cord segments. (Blue: 3U; red: 5U) (a) advanced players; (b) beginner players.

**Figure 2:** Muscle synergy characteristics of advanced and beginner players during jump smash. The vertical axis of motor modules is the normalised per-muscle contribution amplitude (horizontal lines of 0.25, 0.50, 0.75, and 1, respectively), and the scatter indicates the distribution of the trials; the vertical axis of motor primitives is the normalised motor module activation strength (the shaded squares represent significant differences) (a) advanced players; (b) beginner players (left: 3U; right: 5U).

**Figure 3:** Geometrisation characteristics of motor primitives during jump smash for advanced and beginner players (from top to bottom: advanced players, beginners; from left to right: 3U, 5U).

**Figure 4:** Characteristics of synergy index for advanced and beginner players (from top to bottom: 3U, 5U).

**Table 1:** The comparison of the characteristics of the two groups of subjects.

Level	Height (cm)	Weight (kg)	Year	Training period
High-level	178.15 ± 2.51	71.83 ± 7.31	23.39 ± 3.14	>7 years
Low-level	177.64 ± 4.3	74.73 ± 7.9	22.61 ± 2.37	<1 year

**Table 2:** The number and placement of markers in upper-limb segments.

Body segment	Number of markers	Specific placement
Hand	3	First metacarpophalangeal joint; styloid process of radius and ulna
Forearm	3	Lateral 1/3 surface of the forearm; the lateral and medial epicondyle approximating the elbow joint axis
Upper arm	2	Lateral 1/3 surface of the right arm; acromio-clavicular joint
Racket	4	Upper, left, and right sides of the racket; bottom of the racket handle

**Table 3:** The NMF reduction parameters.

Reduction parameters	3U		5U	
	Advanced	Beginner	Advanced	Beginner
Minimum number of synergies	4.47 ± 0.28	4.34 ± 0.41	4.38 ± 0.64	4.26 ± 0.39
Variability accounted for (%)	91 ± 3.7 ^*∗*^	87 ± 4.2	92 ± 2.2 ^*∗*^	89 ± 3.6
Combined synergy (%)	19.2	29.2	18.6	22.6

*Note:* ^*∗*^Indicates a significant difference *P* < 0.05.

## Data Availability

The data that support the finding of this study are available on request from the corresponding author. The data are not publicly available due to privacy or ethical restrictions.
